# Dual-Path Residual “Shrinkage” Network for Side-Scan Sonar Image Classification

**DOI:** 10.1155/2022/6962838

**Published:** 2022-03-24

**Authors:** Fengxue Ruan, Lanxue Dang, Qiang Ge, Qian Zhang, Baojun Qiao, Xianyu Zuo

**Affiliations:** ^1^Henan Key Laboratory of Big Data Analysis and Processing, Henan University, Kaifeng, China; ^2^Henan Province Engineering Research Center of Spatial Information Processing, Henan University, Kaifeng 475004, China; ^3^The Institute of Acoustics of the Chinese Academy of Sciences, Beijing, China

## Abstract

The underwater environment is complicated and changeable and contains many noises, making it difficult to detect a particular object in the underwater environment. At present, the main seabed detection technology explores the seabed environment with sonar equipment. However, the characteristics of underwater sonar imaging (e.g., low contrast, blurred edges, poor texture, and unsatisfactory quality) have serious negative influences on such image classification. Therefore, in this study, we propose a dual-path deep residual “shrinkage” network (DP-DRSN) module, which is a simple and effective neural network attention module that can classify side-scan sonar images. Specifically, the module can extract background and feature texture information of the input feature mapping through different scales (e.g., global average pooling and global max pooling), whereas scale information passes through a two-layer 1 × 1 convolution to increase nonlinearity. This helps realize cross-channel information interaction and information integration simultaneously before outputting threshold parameters in a sigmoid layer. The parameters are then multiplied by the average value of the input feature mapping to obtain a threshold, which is used to denoise the image features using the soft threshold function. The proposed DP-DRSN study provided higher classification accuracy and efficiency than other models. In this way, the feasibility and effectiveness of DP-DRSN in image classification of side-scan sonar are proven.

## 1. Introduction

The continuous improvement of science and technology has deepened human understanding of the ocean. Moreover, frequent marine accidents have given underwater target classification wide application prospects [1, 2]. With the advent of artificial intelligence, deep learning (DL) has made significant progress in the field of image processing. Automatic underwater target classification technology (specifically automatic sonar image target classification) is an essential part of underwater image processing as it relates to ocean exploration, underwater rescue, and other tasks [3, 4]. Owing to the complex and dynamic underwater environment, signal acquisition and transmission, data processing, and other factors often prevent sonar data from being sufficiently accurate, particularly regarding low image contrast, fuzzy edges, and poor textures. Thus, how to improve classification accuracy, speed and reduce the model complexity are the key problems that require urgent solutions.

Presently, many automatic DL-based image classification methods for side-scan sonar (SSS) have been proposed. The main strategy is to extract features through various methods and then use classifiers to learn and classify features. Many feature extraction methods have been proposed for sonar images. Through pixel matrix distribution analysis, the edge and texture information of images are obtained to realize the feature extraction of a target (e.g., a local binary pattern feature extraction algorithm and a histogram of oriented gradient feature extraction algorithm) [5–8]. Mignotte et al. [9] used a Markov random field model, combined with shadow features and shape parameter vectors, to classify sand, pebbles, rocks, ripples, and sand dunes using fuzzy classifiers. Guo et al. [10] proposed an improved gray-level cooccurrence matrix algorithm to classify SSS images using a standard gray-level cooccurrence matrix to extract four texture features, and a support vector machine (SVM) was used to classify the seabed sediment of SSS. Febriawan et al. [11] studied the texture analysis and feature extraction of SSS images with two supervised machine learning methods (SVM and decision tree) and achieved some success in SSS image classification. To further improve classification accuracy, Zhu et al. [12] proposed a sonar image classification method based on principal component analysis and an extreme learning machine; they obtained good stability and improved classification accuracy. Although the above methods effectively improved the classification accuracy to some extent, they only addressed the specific information of sonar images and could not make good use of all feature information. The complexity of the marine environment makes each underwater sonar image different from the seabed. Even image classes have various angles [13], preventing specific extraction methods from being widely used.

Recently, the development of DL technology and its successful application in optical imagery has provided a new solution for sonar imagery. The high-resolution spatial information of seabed sediments plays an essential role in the field of ocean engineering. Therefore, Berthold et al. [14] proposed an automatic sediment classification model for SSS data based on a convolutional neural network (CNN) to infer sediment, achieving good results. Zhu et al. [15] classified sonar images based on shadow and seabed features segmented by the Markov random field-Grabcut algorithm and a CNN model, obtaining better accuracy than a machine learning method. To improve the analysis and utilization rate of feature mapping while reducing the misclassification rate of similar probability categories, Xu et al. [16] used a CNN model to complete their final underwater sonar image classification. Experimental results showed their method could effectively improve the performance of underwater sonar image classification. However, the random initialization of filter weights in a neural network (NN) poses a problem; the model cannot classify underwater targets accurately in sonar images. To solve this problem, Wang et al. [17] proposed an adaptive weighted CNN DL model, generating filter weights with a deep-belief network to adaptively replace randomly trained filter weights. This method can effectively divide sonar images into corresponding seabed categories. Although DL has had a good effect on SSS image classification, the characteristics of SSS images (e.g., low contrast, blurred edges, poor textures, and unsatisfactory image quality) still limit classification accuracy.

To solve the problem based on the residual “shrinkage” network [18], in this study, we propose a dual-path deep residual “shrinkage” network (DP-DRSN) module. Integrating a soft threshold functioninto an attention mechanism will cause unimportant features to be noticed through the mechanism; unimportant features will also be set to zero by the soft threshold, strengthening the ability of the deep CNN (DNN) to extract useful features from noisy signals. Experiments [18] have shown that the residual “shrinkage” network can effectively suppress noise images and improve classification accuracy. Based on the above analysis, the main contributions of this study are as follows:

1. To solve the high noise problem of SSS images, we propose a simple and effective attention module, which eliminates noise-related features by introducing a soft threshold to strengthen the ability of a DNN to extract useful features from noisy signals.
2. A specially designed subnetwork adaptively determines the soft threshold. Because the image features of SSS images are unclear, the subnetwork extracts and aggregates the channel information on the feature map from different scales through global average pooling (GAP) and global max pooling, respectively, so that each channel has its appropriate threshold.
3. Depthwise separable convolution (DSC) is used in the classification model, and the feasibility and effectiveness of DSC in SSS image classification are proven experimentally.

## 2. Model Design

### 2.1. Basic Components

The proposed DP-DRSN has some basic components similar to traditional CNNs (e.g., a convolution layer, rectified linear unit (ReLU) activation function, batch normalization (BN) layer, pooling layer, and sigmoid function). The concepts of these basic components are described in the following.

A convolution layer is the cornerstone of a CNN, and convolution is widely used in the field of image processing. Different convolution kernels can extract different features (such as edge, linearity, and angle). In a deep CNN, some shallow and complex image features can be extracted. In addition, the convolution layer can significantly reduce the number of training parameters, including the most typical 1 × 1 convolution and DSC.

A 1 × 1 convolution can substantially reduce the number of parameters and realize the interaction and integration of cross-channel information, thereby preventing the overfitting phenomenon, which results in relatively high accuracy on a test dataset [19]. The convolution operation between the input feature map and convolution kernel can be expressed as follows:

(1) $$\begin{array}{c} y_{j}=\;\sum_{\;i\in \;M_{j}}x_{i}*k_{ij}+b_{j}, \end{array}$$

where *x*_*i*_ is the *i-*th channel of the input feature maps, *y*_*j*_ is the *j-*th channel of the output feature maps, *k* is the convolution kernel, *b* is the deviation, and *M*_*j*_ is the channel set used to calculate *y*_*j*_. The convolution layer is reused to obtain the output characteristics.

DSC can be decomposed into depthwise and pointwise convolutions [20]. Each channel of the input image is convoluted by depthwise convolution to extract the spatial features of each dimension. Pointwise convolution is a 1 × 1 standard convolution operation on the output feature map, which is used to merge feature maps across diverse channels.

Figure 1 shows the operation process of DSC, given an input image size of *D*_*f*_ × *D*_*f*_ × *M*, where *D*_*f*_ is the height and width of the input image and *M* is the number of channels. Assuming the size of the convolution kernel in the convolution process is *k* × *k*, the size of the output feature mapping after the convolution operation would be *D*_*g*_  × *D*_*g*_ × *M*, where *D*_*g*_ is the height and width of the mapping, and *M* is the number of output feature mapping channels. In pointwise convolution, the size of the convolution kernel is 1  ×  1. The number of channels on each convolution kernel must be the same as the number of input feature mapping channels, allowing a number of convolution kernels *N* to produce output feature mapping of *D*_*g*_ × *D*_*g*_ ×  *N* after convolution.

Introducing an activation function tends to increase the nonlinearity of a CNN model. CNN development has led to the proposition of various activation functions, including sigmoid and ReLU functions. A sigmoid function is a commonly used nonlinear activation function that can transform the continuous real value of the input into output between 0 and 1. It is expressed as follows:

(2) $$\begin{array}{c} y=\;\frac{1}{1+\;e^{-x}}, \end{array}$$

where *x* and *y* are the input and output of a sigmoid activation function, respectively.

Similarly, the ReLU activation function has attracted much attention because it can effectively prevent gradient disappearance while accelerating training speed. It is expressed as follows:

(3) $$\begin{array}{c} y=\max\left(x,0\right), \end{array}$$

where *x* and *y* are the input and output of the ReLU activation function, respectively.

A BN layer is a feature normalization technology that gets inserted into a deep CNN as a trainable network structure [21]. A BN layer is added before the activation function, normalizing the function's input to a fixed distribution (i.e., the mean value is 0 and the standard deviation is 1). During the training process, this layer can solve the problem of changing the data distribution in the middle layer, preventing the gradient from disappearing or exploding while improving the training speed. The process of a BN layer can be expressed using the following formulas:

(4) $$\begin{array}{c} \mu =\;\frac{1}{m}\sum_{i=1}^{m}x_{i},\\ \sigma^{2}=\;\frac{1}{m}\sum_{i=1}^{m}{\left(x_{i}-\mu \right)}^{2},\\ {\hat{x}}_{i}=\;\frac{x_{i}-\;\mu }{\sqrt{\sigma^{2}+\;\varepsilon }},\\ y_{i}=\;\gamma {\hat{x}}_{i}+\;\beta , \end{array}$$

where *x*_*i*_ and *y_i_* represent the input and output of the *i*-th small-batch feature, respectively, *m* is the total number of small-batch characteristics, *y* and *β* are two trainable parameters of distribution scale and shift, respectively, and *ε* is a constant close to 0.

GAP is an operation for calculating the average value of all pixels on the characteristic map of each input channel. It can replace the full connection layer and properly connect categories to their corresponding feature mapping of the last convolution layer. GAP has no parameters (reducing the number of network parameters and preventing overfitting) and can integrate global spatial information; therefore, features learned by a CNN are unaffected by local features. Global max pooling has a similar effect but only focuses on the strongest corresponding part of the feature image, highlighting the foreground information and better retaining the texture features.

### 2.2. Residual Network

ResNet is a super deep CNN with better network performance than a traditional CNN in the fields of image classification, target recognition, and image segmentation [22]. As shown in Figure 2, ResNet's two-layer residual unit comprises double 3 × 3 convolution layers, double BN layers, double ReLU activation functions, and a “shortcut connection.” The input *x* is transmitted to the output as the initial result, and the output result is given by

(5) $$\begin{array}{c} F=W_{2}\delta \left(W_{1}x\right), \end{array}$$

where *W*_1_ and *W*_2_ are the weights of the first and second layers, respectively, and *δ* is the ReLU activation function. This allows *x* to obtain output *y* through the shortcut connection and the second ReLU as follows:

(6) $$\begin{array}{c} y=F\left(x,W_{i}\right)+x. \end{array}$$

When the input and output dimensions need to be changed, a linear transformation *W*_*s*_  can be made for *x* in the shortcut connection.

(7) $$\begin{array}{c} y=F\left(x,W_{i}\right)+W_{s}x. \end{array}$$

To expand into a deeper network model, a three-layer residual block (Figure 3) replaces the two-layer residual block (Figure 2). First, a 1 × 1 convolution is used to reduce the dimension of the number of channels. Then, a 3 × 3 convolution is used to extract features before a 1 × 1 convolution is used to restore the number of channels. This maintains accuracy while reducing the calculation amount. In addition, the original standard 3 × 3 convolution is replaced by DSC to further reduce the model parameters.

In summary, the core of the proposed network module is improved based on the above aspects. Gradual deepening of the network will not cause the parameters to increase significantly, constructing a lightweight residual classification model. The specific network structure will be described in detail in Section 2.3.2.

### 2.3. Model Structure

#### 2.3.1. Theoretical Background

Image denoising often has an STF as the core step [23] on the premise that the function can be used to reduce noise with an eigenvalue lower than the threshold to produce useful information with an eigenvalue greater than the threshold. Generally, the original image is transformed into an unimportant area close to zero before the STF is applied to delete features close to zero. To ensure good image denoising, the key task is to determine a threshold that can properly distinguish useful features from noise while converting noise into near-zero features. However, determining an appropriate threshold requires expertise, and threshold selection has always been a challenging problem [18].

(8) $$\begin{array}{c} y=\;\left\{\begin{array}{cc} x-\;\tau , & x\;>\;\tau ,\\ 0, & \left|x\right|\leq \tau ,\\ x+\tau , & x<-\tau , \end{array}\right) \end{array}$$

where *x* represents the input feature, *y* represents the output feature, and *τ* indicates the threshold. The STF sets near-zero features to 0 and shrinks features far from zero to the threshold.

The denoising process of the STF is shown in Figure 4(a), whereas Figure 4(b) shows the derivative of output to input. The latter shows that the result is either 0 or 1, making it effective for gradient disappearance and explosion problems as well as conducive to the backpropagation of CNNs. The derivative can be expressed as follows:

(9) $$\begin{array}{c} \frac{\partial y}{\partial x}=\left\{\begin{array}{cc} 1, & x\;>\;\tau ,\\ 0, & \left|x\right|\leq \tau ,\\ 1, & x<-\tau . \end{array}\right) \end{array}$$

Setting an appropriate threshold in the process of image denoising is challenging. In addition, the optimal threshold varies according to the image noise. To avoid an error caused by improper threshold setting, the threshold is automatically determined in the DP-DRSN module, which is developed using a deep CNN. The method for determining the DP-DRSN threshold will be introduced in subsequent sections.

#### 2.3.2. DP-DRSN Module

This section describes the DP-DRSN module shown in Figure 5. The difference between the residual networks of Figures 3 and 5 is that the DP-DRSN module has a special subnetwork for determining an appropriate threshold of the STF. In this special subnetwork, an intermediate feature mapping *x* ∈ *R*^*C*×*H*×*W*^ is provided for input, applying the absolute feature map value *x* to pooling layers *M*_GAP_ ∈ *R*^*C*×*l*×*l*^ and *M*_GMP_ ∈ *R*^*C*×*l*×*l*^ to obtain the global compressed feature quantity of the current feature map. The two 1 × 1 convolution layers are then connected. The first convolution layer compresses the number of channels to 1/*S* of its original, reducing the number of model parameters and accelerating the training procedure. In addition, the layer realizes cross-channel information interaction and integration, where *S* is the reduction ratio. The second convolution layer increases the number of channels to its original number and obtains scaling parameters. A sigmoid function is applied at the end of the two-layer convolution to scale the parameters to the range of (0, 1). The sigmoid function is expressed as follows:

(10) $$\begin{array}{c} F\left(z\right)=\;\frac{1}{1+e^{-z}}, \end{array}$$

where *z* is the input of the 1 × 1 convolution in the DP-DRSN module and *F*(*z*) is the scaling parameter output from the sigmoid function. Then, the scaling parameter *α* in Figure 5 can be expressed as follows:

(11) $$\begin{array}{c} F^{\prime }=F\left(M_{\text{GAP}}\left(x\right)\right),\\ F^{\prime \prime }=F\left(M_{\text{GMP}}\left(x\right)\right),\\ \alpha =\;a*F^{\prime }+\;b*F^{\prime \prime }, \end{array}$$

where *a* and *b* are the weights of dual paths and “+” is the element summation symbol.

In the proposed module, the threshold is equal to *α* multiplied by the average of |*x*|, where |*x*| is the absolute value of *x*. The reason for determining the threshold is that it must be positive and cannot be too large, as the latter would cause some useful feature map information to be deleted. When data samples of an SSS image are small and feature information is insufficient, the classification task will be seriously affected. In summary, the threshold can be expressed as follows:

(12) $$\begin{array}{c} \tau =\;\alpha *\text{average}\left|x\right|, \end{array}$$

where *τ* is the threshold.

After the threshold is determined, the STF denoises the input feature mapping *x*, and then *x* is added to the denoised result through the shortcut link. The nonlinearity feature is subsequently added through the ReLU activation function, and its output features are used as the input feature mapping of the next DP-DRSN module.

#### 2.3.3. Classification Model

In this section, we build a CNN model and consider layers 34 and 50 as examples (Figure 6). Detailed parameters are summarized in Table 1. First, the image is subsampled and extracted preliminarily with a 7 × 7 convolution. Second, four residual unit blocks (R1, R2, R3, and R4) are used to continuously extract the spatial context and texture features of the input data. Finally, the adaptive average pooling layer, instead of the full connection layer, is used to fuse the extracted abstract features and make the final classification.

#### 2.3.4. Classification of SSS Image

The characteristics of SSS images make extracting image features difficult. Therefore, as shown in the first layer of the model, a large convolution (7 × 7) is selected to subsample the image and perform preliminary extraction. A larger convolution can extract more complex features and retain as much original image information as possible.

If the convolution kernel is smaller, it is difficult to represent useful features. Experiments have proven that a larger convolution has a better effect in the first layer [24]. R1–R4 modules are stacked with DP-DRSN modules (Figure 5). In each module, a DSC is used to extract the corresponding features, and the threshold is determined by a dual-path attention subnetwork. The STF denoises the extracted features according to the threshold. The reason for this design is that the image features of SSS are unclear, and only a part of the important features can be obtained from a single path. An average pooling layer is more interested in the background information, whereas a max-pooling layer focuses on texture features [25]. A DP-DRSN module extracts the foreground and background information of input feature mapping with different scales, exploiting important features and providing appropriate thresholds. In the three-layer residual block, we place the subnetwork after the 3 × 3 convolution and before the second 1 × 1 convolution. The number of feature mapping channels is reduced through a 1 × 1 convolution in the first layer, whereas the calculation amounts of the subnetwork and STF are reduced in a disguised manner.

To prevent information redundancy, the adaptive average pooling layer (instead of the full connection layer) is used at the end of the model to fuse the extracted feature, further reducing the number of model parameters, alleviating overfitting, and accelerating network convergence [19]. Therefore, the classification model can quickly complete its classification task, reduce noise interference, and improve image classification accuracy. To reiterate, threshold selection is not set by professionals but learned automatically via the network architecture.

## 3. Experimental Settings and Parameter Discussion

### 3.1. Experimental Settings

The workstation configuration used during experimentation is as follows: an Intel® Xeon® E5-1603 v3@2 with an 80 GHz CPU, 32 G internal memory, and NVIDIA Quadro M4000 GPU. We set the dataset batch size to 32 and the learning rate to 0.001. An Adam optimizer was employed to optimize the training parameters, and 200 epochs were performed in each experiment. The proposed model design was actualized with the help of DL frameworks Python 3.6.0 and PyTorch 1.0.0.

The experiments in this section are organized as follows. We analyzed the effects of weights *a* and *b* as well as the scale parameters and network model depth on the classification accuracy in our DP-DRSN. The measurement indices of the experimental results are overall classification accuracy (OA) and average classification accuracy (AA). To ensure accuracy during experimentation, each experiment was performed five times to eliminate the error due to random experimental factors.

In each category of the SSS image dataset, 70% of the images were randomly selected as training samples; the remaining 30% became test samples. The specific sample division of the dataset is shown in Table 2.

### 3.2. Influence of Weights *a* and *b* on Classification Accuracy

Some noise existed in the SSS imagery, which seriously affected the classification effect. Therefore, DP-DRSN was used for denoising. The dual-path weight in the subnetwork structure affected the image classification accuracy. If the proportion of the GAP path is too large, the dual-path module would focus more on the background information. Meanwhile, if the proportion of the global max-pooling path is too large, the module would focus on target object characteristics, highlight the foreground, and extract texture features. Therefore, choosing appropriate proportion parameters is vital. During experimentation, we regarded ResNet50 as the infrastructure and classified the SSS image dataset using a DP-DRSN module. During experimentation, the scaling parameter *S* was initially set to 4. The weight sizes *a* and *b* were set to 1–0 and 0–1, respectively, and their sum was set to 1.

As shown in Figure 7, the classification accuracy varied with the weight ratio. When the weights *a* and *b* were 0.6 and 0.4, respectively, the accuracy was the highest; however, it did not change much between 0.5 and 0.6. In addition, Table 3 shows that the training time did not change much with weight changes, thereby indicating that weight proportion does not affect training times. In the SSS image classification model, we set weights *a* and *b* to 0.6 and 0.4, respectively, as the input of the next experiment.

### 3.3. Effect of Scaling Parameter *S* on Accuracy

In addition to the previously mentioned reasons, the scaling parameter *S* in the DP-DRSN module makes features nonlinear, thereby affecting feature extraction ability and model efficiency. Specifically, small scales prevent decent fitting for a complex correlation between channels while increasing the number of parameters and model calculations. Large scales cause information between channels to be overfitted, yielding information redundancy, which affects accuracy. Therefore, to test the influence of scaling parameters on calculation efficiency and classification accuracy in the SSS image classification model, we selected scaling parameter *S* values of 2, 4, 8, and 16 for experimentation.

As shown in Table 4 and Figure 8, the model had the best accuracy performance when *S* was 4. However, *S* selection had little influence on the training time. In subsequent experimentation, we set *S* to 4 as the input of the next experimental model.

### 3.4. Influence of Network Depth on Classification Accuracy

Network depth directly affects the feature extraction ability of the entire model, with network deepening causing the extraction ability to strengthen. However, too deep a structure can easily yield gradient disappearance, preventing further accuracy improvement. Shallow model structures also do not permit effective FE; therefore, we selected a set of network depth *D* = {10, 18, 34, 50, 71, 101} for experimentation to test the influence of network depth on the classification accuracy of the SSS image dataset. The experimental results are shown in Table 5 and Figure 9. For the SSS image dataset, accuracy first increased and then decreased as the network deepened. When *D* was 34, the classification accuracy of the model reached its peak. Despite strong feature extraction ability, the network was harder to train on smaller datasets, making the model unstable and easy to oscillate. In summary, the 34-layer network produced the highest accuracy and a relatively short training time. Therefore, we chose the 34-layer network as the infrastructure for experimentation.

## 4. Results and Discussion

To verify the classification performance of the proposed classification model, we selected typical recent classification models of SSS images, such as VGG16 [26], ResNet34 [22], ResNet50 [22], DenseNet [16], MobileNet [27], and ShuffleNet [28]. Specifically, VGG16 is a typical model of DL applied to SSS image classification. With the further development of the network, ResNet34 and ResNet50 with stronger feature extraction ability were gradually applied to the classification of SSS images. Owing to the small amount of SSS image data, people prefer to use lightweight networks, such as DenseNet, MobileNet, and ShuffleNet, for classification.

In addition, to further measure the performance of the proposed classification model, we performed a more detailed comparative experiment using effective attention mechanisms in the classification network. These were the squeeze and excitation (SE) module [29], convolutional block attention module (CBAM) [30], and deep residual shrinkage network with channelwise thresholds (RSBU-CW) [18]. Further, an Std-CNN was established using standard convolution based on DP-DRSN. To ensure experimental fairness, each group was tested five times. The parameters of the proposed classification model were determined in Section 3. OA, AA, and the kappa coefficient were used as evaluation indices, with AA being expressed in the form of “average results of five experiments plus standard deviation.”

A detailed comparison was made between DP-DRSN and Std-CNN to verify the feasibility and effectiveness of DSC in a SSS image dataset.

### 4.1. Comparison with Other Methods

The classification results are shown in Table 6. It can be seen from the results that, among all classification models, the classification accuracy (OA; AA) of the proposed model is better than that of other classification models. Particularly, compared with VGG16, the proposed model is 7.59% higher. Besides, it is 3.57% and 4.47% higher than deep CNNs (ResNet34; ResNet50) and about 1.34% higher than lightweight networks (DenseNet, MobileNet, and ShuffleNet). Obviously, the classification accuracy of the deep network model and lightweight network model is lower than that of the proposed model. This means that the noise in the SSS image has a negative impact on the classification, and the features extracted only by the model are not enough to achieve higher classification accuracy. It should be pointed out that the training time of the model proposed in this paper is slightly longer than that of the lightweight network, but the gap is not obvious. The results show that the denoising method based on the attention mechanism proposed in this paper can improve the classification accuracy and efficiency to a certain extent in the SSS image task.

In order to further verify the performance of this method, based on ResNet34 and ResNet50, we make a detailed comparison with other attention mechanisms which have good results in other classifications. The results are shown in Table 7. Both infrastructures show that the classification accuracy of the proposed model was higher than that of the other classification models, indicating our proposed module performed well. Specifically, the OA of the proposed model was ∼4.5%, 2.23%, and 1.79% higher than that of ResNet34, channel attention module (SE), and CBAM, respectively. In addition, the AA and kappa coefficients were better than those of the other classification models. In ResNet34, the performance (OA, AA, and kappa) of Std-CNN was superior, proving that DP-DRSN is more suitable for SSS image classification than other modules. In ResNet50, the classification accuracy of the proposed model also had a significant improvement (∼1.80% higher than other models); however, the ability of Std-CNN was slightly inferior due to the network being relatively deep and possessing numerous parameters. Similarly, DP-DRSN is relatively complex and difficult to train for small sample datasets. However, this situation can be significantly alleviated using DSC. We perform a detailed analysis in Section 4.2.

In addition, the AA of the RSBU-CW is better than SE and CBAM, and the standard deviation is lower. This shows that the classification accuracy and model stability using only attention modules (SE; CBAM) are lower than those using the residual “shrinkage” network module (RSBU-CW). The RSBU-CW module can eliminate image noise at a certain level and improve classification accuracy. However, it should be pointed out that, due to the characteristics of SSS image, such as fuzzy edge, low contrast, and unsatisfactory image features, RSBU-CW has poor feature extraction ability when extracting features from a single scale to determine the threshold and cannot give an appropriate threshold, which results in limited improvement of model classification accuracy. In contrast, the proposed model extracts image features from different scales and is better in determining thresholds. As can be seen from Table 6, OA and AA of the proposed model are superior to the RSBU-CW module, which are 1.79% and 1.52% higher, respectively. This proves that the proposed model has good classification performance on the SSS dataset.

In addition, the AA of the RSBU-CW module was better than that of the SE module and CBAM, with a lower standard deviation, indicating that the classification accuracy and model stability of attention modules (SE and CBAM) were lower than those of a residual shrinkage network module (RSBU-CW). The RSBU-CW module can eliminate image noise at a certain level and improve classification accuracy. However, owing to the characteristics of SSS imagery (e.g., fuzzy edges, low contrast, and unsatisfactory image features), RSBU-CW has poor feature extraction ability when extracting features from a single scale to determine the threshold. It also cannot provide an appropriate threshold, limiting model classification accuracy improvement. By contrast, the proposed model can extract image features from different scales and is better in determining thresholds. Table 7 shows that the OA and AA of the proposed model are 1.79% and 1.52%, respectively, higher than those of the RSBU-CW module, indicating that the proposed model has good classification performance with the dataset.

To further verify the performance, we present a confusion matrix for each model based on the ResNet34 structure (Table 8). Compared with other models (SE, CABM, and RSBU-CW), the proposed model slightly increased the number of correct predictions for three image types: aircraft, seafloor, and shipwreck. Although the number was relatively small, it provided a significant improvement for fewer numbers of SSS image samples. While there was no improvement in the seafloor category compared with the SE module, four more images were predicted correctly in the aircraft category, especially when the total number of aircraft in the test set was 18 images, demonstrating a particularly objective improvement. However, in the category of drowning victims, the proposed model's performance was slightly insufficient, registering fewer correct images less than CABM and RSBU-CW. This may be due to the proposed model being relatively complex in structure and the small number of drowning victims preventing adequate network parameter training. This would cause discretely inferior classification performance. In addition, all models possessed a large error rate in the aircraft category due to the target objects of some aircraft images being too small or incomplete. Accuracy could be improved by redefining the size of target objects [31].

In Table 8, the figures in blue are the predicted categories that match the true categories, whereas those in red are the prediction errors.

Figure 10 shows the visualization results of the first 12 channels in the first convolution layer of each model, as well as the original SSS image. The original image features are fuzzy, and there is noise interference on the feature maps without the use of an attention module for classification (Figure 10(a)). Although the attention module networks (SE and CBAM) can notice the target object well, they still have noise interference problems (Figures 10(b) and 10(c)).  Figure 10(d) shows that although RSBU-CW eliminates the influence of noise at a certain level, the background features are clearer and the target features are more three-dimensional. However, the edge of the target object was not handled well, the edge features are slightly blurred, and noise interference still exists. The proposed model can overcome these shortcomings.  Figure 10(e) indicates that the proposed model largely eliminated noise interference, thereby producing a clear and smooth background, three-dimensional target features, and clearer edge features. This demonstrates the strong feature extraction ability of the proposed model via intuitive comparison of the channel feature maps, further proving that the proposed model has good performance on the SSS dataset.

To prove that the proposed model also has a good classification effect in the category of drowning victims, we set the number of drowning victim samples in the test set to *S* = {5, 10, 15, 18} (the total number of drowning victims was 18), and the data came from the training set. In addition, simulated SSS images [31] were added to the training set. For experimental fairness, we performed five experiments with each group, selected the batch with the highest accuracy, and obtained the number of correct and incorrect drowning victim predictions to evaluate the classification performance of the proposed model in the category of drowning victims.

As shown in Figure 11, for small sample numbers (*S* = 5 and 10), all models possessed similar classification ability because simulated SSS images improved model learning ability and significantly alleviated the problem of feature representation ability being limited due to training parameters.  Table 9 and Figure 11 show that, as the number of samples increased, the number of correct classifications of the proposed model increased, despite the classification accuracy of other models gradually decreasing. To a certain extent, this indicates that the addition of simulated images alleviates the proposed model's classification problem but is insufficient to support the classification of more test samples by the model. However, when *S* = 15, the proposed model's accuracy improved well beyond the other models, indicating that the proposed model had a strong learning ability. When *S* = 18 (i.e., no real SSS images in the training set), the number of correct predictions provided by CBAM and the proposed model did not increase as the number of training samples increased. Even CBAM had a problem with decreasing correct predictions. This may be due to the simulated images retaining the main contour of the target object and conforming to the distribution of the real image [32]. A gap remained between the simulated and real images in the spatial context, background, and noise information. When no real images were part of the training dataset, some deviations in the training process of both CBAM (concentrating on spatial information) and the proposed model (focusing on foreground and background information) affected the classification accuracy to a certain extent. Despite being negatively affected, the classification ability of the proposed model was equivalent to that of RSBU-CW. Experimental results showed that the proposed model's classification ability was not inferior to other models while maintaining strong learning ability.

In the last part of the experimentation, we compared ResNet34 and ResNet34 with SE, ResNet34 with CBAM, ResNet34 with RSBU-CW, and the proposed model from three aspects: floating-point operations per second (FLOPs), the number of model parameters, and training time. As shown in Figure 12, the model parameters for our proposal were much lower than those of other models. Figure 12 and Table 10 indicate that although the number of parameters in the proposed model was small, its training time was not much lower than that of other models as well as even higher than that of ResNet34. The main reason for this is that model training times are determined by the number of model parameters and the model's structure. Our model's structure is more complicated; however, we can reduce parameters through DSC, which makes it easier to train a model on small sample datasets and improve classification accuracy, despite our model's complex structure affecting training speed.

In addition, to analyze the complexity of the model, a widely used measure is the number of FLOPs during model inference. It is an indirect measure and an approximate estimate of the direct measure we really care about, such as speed or delay. The proposed model has the lowest number of FLOPs due to the fact that DSC reduces the number of model parameters and makes the model have a lower computation cost. In summary, the proposed model has high accuracy and is better than other models in terms of the number of parameters, training time, and FLOPs.

### 4.2. Analysis of DSC Effectiveness

In this section, we perform a detailed comparison between Std-CNN and DP-DRSN to verify the feasibility and effectiveness of the DSC method for SSS images.  Table 11 presents the OA, AA, kappa coefficient, FLOPs, number of model parameters, and training times of the two models. The DP-DRSN had higher OA, AA, and kappa coefficient values. Specifically, considering the matching hyperparameters, all results for the DP-DRSN exceeded those of Std-CNN, especially in the ResNet50 architecture. In addition, the training times of the DP-DRSN were lower than those of Std-CNN.

Model complexity and computation are also essential factors.  Figure 13 shows the training parameters and FLOPs of Std-CNN and DP-DRSN under different NNs. The training parameters and FLOPs of Std-CNN were higher than those of DP-DRSN in the same configuration. Specifically, the FLOPs of Std-CNN were 3.674 and 4.114 G, which were twice those of DP-DRSN. Moreover, the Std-CNN training parameters were 22.428 and 26.188 M, which are also about twice those of DP-DRSN. According to the above analysis, the proposed model achieved better results than Std-CNN when classifying the SSS dataset, improving classification accuracy (OA, AA, and kappa) and shortening training times while outperforming Std-CNN regarding model complexity and computation. These results sufficiently prove that DSC is feasible for SSS image classification.

Although the proposed model improves the classification accuracy to a certain extent, there are still many image classification errors. The use of deep separable convolution reduces the model parameters to a certain degree; however, when there are few training samples, the model cannot be fully trained, cannot converge, has poor generalization ability, and is prone to misclassification, especially in the aircraft category. The reason is that the aircraft structure is complex, and feature extraction is not easy, especially when there are few training samples and insufficient model training, which further increases the difficulty of feature extraction. In future work, aiming at this problem, we will expand the dataset and use dense links combined with an attention mechanism to classify SSS images.

## 5. Conclusions

In this study, we proposed and discussed a DP-DRSN attention module that combined a ResNet architecture with DSC to construct an SSS classification model. During experimentation, we analyzed the influence of the weight ratio of the two paths in the DP-DRSN module, scaling parameters, and network depth on classification accuracy. Then, we compared the proposed model with other classification models using set parameters. Results showed the proposed model not only ensured high classification accuracy but also significantly reduced the number of parameters and improved the classification speed. In addition, the proposed model possessed a strong feature extraction ability for an SSS image dataset containing high noise and fuzzy edge features. We also explored the proposed model's accuracy using standard convolution and DSC while changing the number of parameters and FLOPs in the SSS images. The results showed that DSC had feasible application to the small sample dataset of SSS. Compared with Std-CNN, the proposed model had better accuracy and performance, making it better for performing rapid rescue tasks.

## Figures and Tables

**Figure 1:** Depthwise separable convolution.

**Figure 2:** Two-layer residual block.

**Figure 3:** Three-layer residual block.

**Figure 4:** (a) Soft threshold function and (b) its derivative.

**Figure 5:** Structure of DP-DRSN module; (*K*) is the size of the convolution kernel.

**Figure 6:** Classification model of dual-path residual “shrinkage” network.

**Figure 7:** Influence of different weight ratios on accuracy.

**Figure 8:** Influence of different scaling parameters *S* on classification accuracy.

**Figure 9:** Influence of network depth on classification accuracy.

**Figure 10:** The first 12 channel feature maps in the first convolution layer of (a) ResNet34, (b) SE, (c) CBAM, (d) RSBU-CW, and (e) proposed model. (f) Original side-scan sonar image.

**Figure 11:** Classification accuracy of each model in the drowning victim category.

**Figure 12:** Comparison of parameter quantity of each model.

**Figure 13:** Comparison of (a) FLOPs and (b) parameter number of the proposed model with DSC and standard convolution.

**Table 1:** Detailed configuration of the 34- and 50-layer network infrastructure frameworks.

Layer	Output size	Kernel size		Module numbers
		Residual block (two)	Residual block (tree)	
Conv1	112 × 112	7 × 7 × 64 (Conv) 3 × 3 (max pooling)		

R1	56 × 56	3 × 3 × 64 (Conv) 3 × 3 × 64 (DS-Conv)	1 × 1 × 64 (Conv) 3 × 3 × 64 (DS-Conv) 1 × 1 × 256 (Conv)	3

R2	28 × 28	3 × 3 × 128 (Conv) 3 × 3 × 128 (DS-Conv)	1 × 1 × 128 (Conv) 3 × 3 × 128 (DS-Conv) 1 × 1 × 512 (Conv)	4

R3	14 × 14	3 × 3 × 256 (Conv) 3 × 3 × 256 (DS-Conv)	1 × 1 × 256 (Conv) 1 × 1 × 256 (DS-Conv) 1 × 1 × 1024 (Conv)	6

R4	7 × 7	3 × 3 × 512 (Conv) 3 × 3 × 512 (DS-Conv)	1 × 1 × 512 (Conv) 3 × 3 × 512 (DS-Conv) 1 × 1 × 2048 (Conv)	3

GAP	1 × 1			

**Table 2:** Detailed information of the SSS image dataset.

Class	Total	Train	Test
Drowning victim	18	13	5
Aircraft	60	42	18
Seafloor	289	203	86
Shipwreck	385	270	115
Total	752	528	224

**Table 3:** Classification accuracy under different proportions of weights *a* and *b*.

*a* and *b*	OA (%)	AA (%)	Time (s)
1 and 0	93.75 ± 0.45	93.66 ± 0.52	7335
0.9 and 0.1	93.75 ± 0.45	93.39 ± 0.44	7243
0.8 and 0.2	93.75 ± 0.45	93.03 ± 0.67	7336
0.7 and 0.3	93.30 ± 0.45	93.48 ± 0.36	7386
0.6 and 0.4	94.64 ± 0.45	94.10 ± 0.59	7416
0.5 and 0.5	94.20 ± 0.45	94.01 ± 0.45	7335
0.4 and 0.6	93.30 ± 0.45	93.48 ± 0.25	7420
0.3 and 0.7	93.75 ± 0.45	93.52 ± 0.46	7290
0.2 and 0.8	93.75 ± 0.45	93.57 ± 0.67	7100
0.1 and 0.9	93.75 ± 0.45	93.39 ± 0.33	7230
0 and 1	93.75 ± 0.45	93.48 ± 0.46	7155

**Table 4:** Effects of scaling parameter on accuracy.

*S*	OA (%)	AA (%)	Time (s)
2	93.30 ± 0.45	93.03 ± 0.61	7898 ± 219
4	94.75 ± 0.90	94.10 ± 0.59	7335 ± 143
8	93.75 ± 0.45	93.66 ± 0.44	7732 ± 17
16	93.75 ± 0.45	93.57 ± 0.46	7535 ± 168

**Table 5:** Influence of network depth on classification accuracy.

S	OA (%)	AA (%)	Time (s)
10	92.86 ± 0.45	92.94 ± 0.33	3132 ± 92
18	93.30 ± 0.45	93.48 ± 0.36	3436 ± 83
34	95.09 ± 0.45	95.0 ± 0.44	5110 ± 79
50	94.64 ± 0.45	94.10 ± 0.59	7386 ± 152
71	93.30 ± 0.45	93.21 ±0.52	10272 ± 192
101	92.86 ± 0.45	92.68 ± 0.22	14068 ± 241

**Table 6:** Classification performance of each model.

Model	OA (%)	AA (%)	Time (s)
VGG16	87.50 ± 0.45	87.50	14599
ResNet34	91.52 ± 0.45	91.52	4690
ResNet50	90.62 ± 0.90	90.71	9499
DenseNet	93.75 ± 090	93.40	7568
MobileNet	93.30 ± 0.45	93.13	4840
ShuffleNet	94.20 ± 090	94.29	4509
Proposed	95.09 ± 0.45	95.0	5110

**Table 7:** Classification performance of each model.

Model	OA (%)	AA (%)	Kappa × 100
ResNet34 + SE	92.86 ± 0.45	92.94 ± 0.35	87.38 ± 0.75
ResNet34+CBAM	93.30 ± 0.45	93.21 ± 0.44	88.28 ± 0.05
ResNet34+RSBU-CW	93.30 ± 0.45	93.48 ± 0.22	89.03 ± 0.82
Std-CNN	94.64 ± 0.45	94.28 ± 0.63	91.29 ± 0.26
Proposed	95.09 ± 0.45	95.0 ± 0.44	92.14 ± 0.13
ResNet50 + SE	92.41 ± 0.45	92.41 ± 0.49	85.92 ± 1.00
ResNet50 + CBAM	92.86 ± 0.45	92.86±0.28	87.21±0.14
ResNet50 + RSBU-CW	93.30 ± 0.45	93.21 ± 0.52	87.30 ± 0.11
Std-CNN	92.86 ± 0.45	92.76±0.33	86.51±0.23
Proposed	94.64 ± 0.45	94.10 ± 0.59	90.60 ± 0.16

**Table 8:** Confusion matrix of each model.

Model	True class	Predicted class			
		Drowning victims	Aircraft	Seafloor	Shipwreck
ResNet34 + SE	Drowning victim	4	0	0	1
	Aircraft	0	7	2	9
	Seafloor	0	1	85	0
	Shipwreck	1	1	1	112

ResNet34 + CBAM	Drowning victim	5	0	0	0
	Aircraft	0	9	0	9
	Seafloor	0	0	84	2
	Shipwreck	1	3	0	111

ResNet34 + RSBU-CW	Drowning victim	5	0	0	0
	Aircraft	0	10	0	8
	Seafloor	0	0	83	3
	Shipwreck	1	1	1	112

Proposed	Drowning victim	4	0	0	1
	Aircraft	0	11	0	7
	Seafloor	0	0	85	1
	Shipwreck	0	1	0	114

**Table 9:** Number of correct and incorrect predictions of drowning victim category when the number of samples is 5, 10, 15, and 18.

Number of samples	Predicted class	Model			
		ResNet34 + SE	ResNet34 + CBAM	ResNet34 + RSBU-CW	Proposed
5	Drowning victim	5	5	5	5
	Aircraft	0	0	0	0
	Seafloor	0	0	0	0
	Shipwreck	0	0	0	0

10	Drowning victim	9	9	9	9
	Aircraft	0	0	0	0
	Seafloor	0	0	0	0
	Shipwreck	1	1	1	1

15	Drowning victim	12	11	12	14
	Aircraft	0	1	1	0
	Seafloor	0	0	0	0
	Shipwreck	3	3	2	1

18	Drowning victim	13	10	14	14
	Aircraft	0	6	0	1
	Seafloor	1	0	0	0
	Shipwreck	4	2	4	3

**Table 10:** FLOPs and training time of each model.

		SE	CBAM	RSBU-CW	Proposed
ResNet34	FLOPs (G)	3.671	3.674	3.675	1.837
	Time (s)	5124 ± 152	5300 ± 164	5495 ± 220	5110 ± 79

ResNet50	FLOPs (G)	4.112	4.115	4.115	2.227
	Time (s)	7562 ± 150	7583 ± 188	7683 ± 116	7335 ± 143

**Table 11:** Classification performance of the proposed model with DSC and standard convolution.

Model		OA (%)	AA (%)	Kappa × 100	Time (s)
ResNet34	Std-CNN	94.64 ± 0.45	94.28 ± 0.63	91.29 ± 0.26	5441 ± 110
	DP-DRSN	95.09 ± 0.45	95.0 ± 0.44	92.14 ± 0.13	5110 ± 79

ResNet50	Std-CNN	92.86 ± 0.45	92.76 ± 0.33	86.51 ± 0.23	9257 ± 168
	DP-DRSN	94.64 ± 0.45	94.10 ± 0.87	90.60 ± 0.16	7335± 143

## Data Availability

Data cannot be made public.
